RETRACTED

# National database study on the use of long‐acting antipsychotic injections and hospital readmission proportions in patients with schizophrenia in Japan

**DOI:** 10.1111/pcn.12970

**Published:** 2020-02-03

**Authors:** Masato Usuki, Yuhei Kamiura, Ryo Okubo, Yoshio Yamanouchi

**Affiliations:** ^1^ Department of Mental Health Policy National Institute of Mental Health, National Center of Neurology and Psychiatry Tokyo Japan; ^2^ Department of Medical Affairs Otsuka Pharmaceutical Co., Ltd. Tokyo Japan; ^3^ Department of Clinical Epidemiology Translational Medical Center, National Center of Neurology and Psychiatry Tokyo Japan

**Keywords:** antipsychotic agents, injections, Japan, patient readmission, schizophrenia

## Abstract

**Aim:**

It is important to investigate the current prescription status and clinical outcomes of patients with schizophrenia receiving long‐acting antipsychotic injections. We aimed to determine the prescription proportion of long‐acting antipsychotic injections and hospital readmission proportions of patients with schizophrenia in Japan.

**Methods:**

An open dataset was created using data from the National Database of Health Insurance Claims and Specific Health Checkups of Japan. Patient records with the term ‘schizophrenia’ were included. In Analysis 1, antipsychotic prescription proportions were determined for outpatients who had visited psychiatric facilities between 1 February 2015 and 31 March 2017. In Analysis 2, patients who had been discharged from a psychiatric facility and had received a long‐acting antipsychotic injection prescription within 90 days after initial discharge were selected; then, their readmission proportion was examined for 365 days after the initial discharge.

**Results:**

The long‐acting antipsychotic injection prescription proportion was 3.5% for outpatients with schizophrenia receiving antipsychotics. The readmission proportion was 41.0% in the entire patient population, 36.2% in patients receiving typical long‐acting antipsychotic injections alone, and 23.5% in patients receiving atypical long‐acting antipsychotic injections alone.

**Conclusion:**

Long‐acting antipsychotic injections are not yet widely used in Japan. The readmission proportion was lower in the patients receiving atypical than typical long‐acting antipsychotics injections. The results may provide important basic information to develop new future research questions but should be interpreted with caution because generalizability may be limited by the use of aggregated data and the data structure of the database used.

Schizophrenia is a chronic disease, and most patients experience relapses even when symptoms have previously been alleviated by antipsychotic treatment.^1^ The high rate of relapse is a serious issue worldwide and repeated relapses decrease social functioning in this population.^2^ Antipsychotic treatment discontinuation is the factor most strongly associated with relapse of schizophrenia according to a systematic review and a prospective study.^1^, ^3^ This indicates that improving long‐term drug adherence is an urgent issue that needs to be addressed in any therapeutic strategy for this disorder.^1^, ^4^, ^5^

Long‐acting antipsychotics injections (LAIs) have become widely used around the world.^6^ They are recommended as a treatment option for patients who prefer this route of administration in various schizophrenia treatment guidelines such as the United Kingdom National Institute for Health and Care Excellence^7^ and the Maudsley Prescribing Guidelines in Psychiatry (13th edition).^8^ Some LAIs have also been recommended by the World Federation of Societies of Biological Psychiatry Guidelines for Biological Treatment of Schizophrenia.^9^

RETRACTED

Prevention of relapse decreases readmission proportions and therefore decreases time spent in a psychiatric facility. The Ministry of Health, Labour and Welfare (MHLW) of Japan has produced publications entitled ‘Vision for Reform of Mental Health Care and Welfare’^10^ and ‘Guidelines to Securing High Quality and Appropriate Healthcare for Patients with Psychiatric Disorders’,^11^ which emphasize the importance of early discharge from hospital and local community integration for patients with acute‐stage schizophrenia.

LAIs may help prevent readmission and extend time spent in the community, and were found to be marked superior to oral antipsychotics (OAPs) in preventing hospitalization according to a meta‐analysis of mirror‐image studies.^12^ In addition, Kishimoto and colleagues found in a meta‐analysis of cohort studies that hospitalization rate and all‐cause discontinuations were significantly lower when using LAIs compared with OAPs.^13^ Taking into account the efficacy of LAIs compared with oral agents, the aforementioned guidelines, and adherence issues, it is of great clinical significance to consider an LAI regimen.

Several studies have investigated LAI usage in Japan, and found that LAIs have not been widely adopted by Japanese psychiatrists. Tanaka and Fujii reported that the LAI prescription proportion at Yamanashi Prefectural Kita Hospital was 15.6%.^14^ Shibata and colleagues recruited 25 346 schizophrenia patients (163 facilities) in 2010 and 22 000 schizophrenia patients (148 facilities) in 2011 and found that the LAI prescription proportion was 7.6%–8.2%.^15^ However, Barnes *et al*. reported that LAIs were prescribed in 36% of 1616 assertive outreach team patients with schizophrenia in the UK and Humberstone *et al*. reported that LAIs were prescribed in 23.3% of 3178 outpatients who received antipsychotics in Auckland, New Zealand.^16^, ^17^ The proportion of LAI prescriptions appears to be lower in Japan than in other countries, but these figures cannot simply be compared because of differences in study design and eligibility criteria among the studies.

RETRACTED

It is also clinically important to determine regional variations in the LAI prescriptions proportion. For example, Covell *et al*. analyzed antipsychotics prescriptions among outpatients with schizophrenia spectrum disorders in Connecticut, USA and reported an LAI prescription proportion of 28%.^18^ In contrast, a study involving patients with schizophrenia in California found an LAI prescription proportion of 5.6%.^19^ However, these figures cannot simply be compared because each study had different study designs and methods of data analysis.

To realize the MHLW's goal of early discharge and community integration for inpatients with acute schizophrenia, it is important to understand the conditions that lead to re‐hospitalization. Cheung and colleagues studied re‐hospitalization and emergency department visit rates using the Diagnostic Procedure Combination database. They found that both of these rates decreased more with LAIs prescriptions than with OAP prescriptions. They also found that re‐hospitalization and emergency department visit rates decreased more with typical and atypical LAI prescriptions than with OAP prescriptions, but this decrease was not statistically significant.^20^ However, they did not compare the rates between typical or atypical LAI prescriptions. Their data source was also limited to only hospitals listed in the Diagnostic Procedure Combination database. No nationwide study has comprehensively investigated the types of LAIs prescribed and the rate of relapse in patients with schizophrenia in an outpatient setting, where the choice of LAI is important due to adherence issues.

Against this background, we conducted this nationwide survey investigating LAI prescriptions and readmission proportions among outpatients with schizophrenia in Japan—both nationwide and in individual prefectures—by applying the same analytical approach to data collected during the same period. The purpose of this study was to investigate the current status of LAI prescriptions for outpatients with schizophrenia in Japan and to investigate the readmission proportion and the current status of LAI prescriptions for outpatients with schizophrenia after psychiatric hospitalization.

## Methods

### Data source

The National Database of Health Insurance Claims and Specific Health Check‐ups of Japan (NDB) is operated by the MHLW.^21^ It contains the claims data of the commonly used national health insurance system to which most Japanese people subscribe and which permits low out‐of‐pocket medical expenses for patients. Since 2011, it has been possible for researchers to use the NDB for identifying accurate evidence on which promotion of policies may be based, with the aim of improving the quality of medical services, or for conducting analysis and research that are useful for these policies, and for advancing academic research. The NDB covers almost all patients who have received medical care services under the universal health insurance system, but does not include medical services that are not covered under this system.^22^ We used datasets from a policy research group's study entitled ‘Policy research for promoting functional reinforcement of the psychiatric care provision system’ to extract data in line with our objectives and to create a separate dataset for our retrospective study.

RETRACTED

The policy research group started in 2016 to establish various datasets useful for policy making and was supported by an MHLW research grant,^23^ under contract with the MHLW and complies with the ‘Guidelines on Supply of Insurance Bill Information and Information on Specific Health Checkups’. These aggregated datasets are not publicly available, but publication of such data may be permitted by the MHLW if doing so is in the public interest. YY, MU and YK are authors of this study but only YY and MU are members of the policy research group. Together, these three authors discussed the present study's design, then YY and MU developed the dataset for this study by extracting data from the policy research group's datasets. MU and YK then selected patient data that met the inclusion criteria from the dataset for this study. YK did not have direct access to aggregated data and the dataset for this study did not include patient‐specific information. The dataset for this study contained data for the period from 1 February 2015 to 31 March 2017.

The MHLW has approved public access to our dataset, which is available at https://www.ncnp.go.jp/nimh/seisaku/study/analysis/assets/0002.xlsx.

### Study design and study period

In this study, an NDB‐derived dataset was created to investigate the LAI prescription status in outpatients with schizophrenia and to determine the readmission proportions of previously discharged patients according to whether they were prescribed typical or atypical LAI treatment.

The study period is illustrated in Figure 1.

**Figure 1:** Study design. (a) Analysis 1. (b) Analysis 2.

RETRACTED

This study involved two analyses of outpatients with schizophrenia who were prescribed antipsychotic drugs. Analysis 1 examined the LAI prescription proportion, and Analysis 2 examined the readmission proportion after discharge. The index date for inclusion in Analysis 1 was the date of the first antipsychotic prescription during the evaluation period. For Analysis 2, the index date for inclusion was the date of the first LAI prescription within 90 days after discharge from a psychiatric facility.

Patients who met the inclusion criteria were included in the study. We did not set the exclusion sequences, enrollment windows, and enrollment gaps for the dataset, which were decided by the policy research group. The inclusion and exclusion windows for the present study's dataset were defined as between 1 February 2015 and 29 June 2016.

### Patient selection

Subjects in Analysis 1 and Analysis 2 were outpatients prescribed antipsychotic drugs. We used the list of antipsychotic drugs approved in Japan and classified them according to the Drug Master of the Clinical Care Fee Information Supply Service (http://www.iryohoken.go.jp/shinryohoshu/downloadMenu), which is provided by the Health Insurance Bureau of the MHLW. This list was used to identify antipsychotics in the policy research group's dataset. Antipsychotics were classified as typical or atypical based on atypical antipsychotics listed as additional items and as LAIs or non‐LAIs based on the dosage form (Table SS1, Code D4). We excluded chlorpromazine‐promethazine‐phenobarbital, reserpine, and tiapride because these drugs are not usually used to treat patients with schizophrenia in the clinical setting. Also, in Japan, chlorpromazine‐promethazine‐phenobarbital is used for sedation and hypnosis, not for the treatment of schizophrenia. Reserpine is mainly used to treat hypertension and tiapride is mainly used to treat sequelae of cerebral infarction. Their use is considered off‐label for schizophrenia. Prescriptions were additionally included, except for prescription of as‐needed administration of antipsychotics.

Patients with schizophrenia definitively diagnosed in March 2017 or earlier were also included. Patients with a suspected diagnosis were excluded.

In Analysis 1, outpatients with schizophrenia receiving antipsychotics met the following criteria: (1) Prescribed antipsychotics based on diagnosis code F20–F29 according to the International Classification of Diseases, 10th Revision (ICD‐10; Table SS1, Code C7) and whose fee for outpatient psychiatric care was calculated during the evaluation period. (2) Prescribed antipsychotics appearing in the ‘Matters Regarding Listing in the Ethical Drug Price List’^24^ published in Japan (Table SS1, Code C7).

RETRACTED

In Analysis 2, patients were classified into one of six groups based on prescriptions during the time from discharge to readmission or at the end of the follow‐up period if not readmitted. The six prescription groups were (1) prescribed only typical LAI, (2) prescribed only atypical LAI, (3) prescribed typical and atypical LAI, (4) prescribed typical LAI and non‐LAI, (5) prescribed atypical LAI and non‐LAI, and (6) prescribed typical LAI, atypical LAI, and non‐LAI.

Furthermore, in Analysis 2, patients who received LAI prescriptions within 90 days after discharge from a psychiatric facility met the following criteria: (i) hospitalized for schizophrenia and discharged from a psychiatric facility between 1 February 2015 and 31 March 2016 and before discharge received treatment based on diagnosis code F20–F29 according to ICD‐10 (Table SS1, Code C7), and (ii) received an LAI outpatient prescription within 90 days after discharge (Table SS1, Code C7).

### Exposure and follow‐up

Subjects were outpatients in both Analysis 1 and Analysis 2. For Analysis 2, exposure was defined as LAI prescription within the first 90 days after discharge from a psychiatric facility and the follow‐up period was 365 days after discharge. It was necessary to include patients who received LAIs during continuous medical treatment after discharge. The Japanese national health insurance system regards such patients as new patients if they have not visited a hospital within 90 days after discharge. Therefore, we regarded patients with an LAI prescription within 90 days after discharge as receiving continuous medical treatment from discharge and included them in our study.

The 29 antipsychotics that are currently used to treat schizophrenia patients in Japan were selected and classified as either typical or atypical antipsychotics and as either LAI or non‐LAI according to the formulation described in the claims database (Table SS2).

### Outcomes

In Analysis 1, the event date was defined as occurring between 1 February 2015 and 31 March 2016. The proportion of patients who had received LAIs was defined as the proportion of outpatients who had been assigned a drug code corresponding to LAIs and who met the inclusion criteria (Table SS1, Code D4). When calculating the antipsychotics prescription proportion in each prefecture, if the same patient had received another prescription from another prefecture, then that prescription was counted separately.

In Analysis 2, the readmission date was defined as the date of the first psychiatric hospitalization within 365 days after discharge from a psychiatric facility (Table SS1, Code F1).

RETRACTED

Furthermore, in Analysis 2, the readmission proportion was defined for each prescription group as the number of patients readmitted within 365 days after discharge out of the total number of patients in the group (Table SS1, Code F2).

### Ethical considerations

Informed consent could be waived because only anonymous and aggregated data were used. Furthermore, according to the Japanese Ethical Guidelines for Medical and Health Research Involving Human Subjects, the institutional review board did not need to be informed of our research because all data were based solely on summary tables (i.e. secondary use of a database). In addition, our study was approved in advance by the committee for commissioned joint research of the National Center of Neurology and Psychiatry in Japan.

### Statistical analysis

In Analysis 1, summary tables from the policy research group were used to obtain the number of patients who had received antipsychotics. In Analysis 2, summary tables from the policy research group were used to obtain the number of patients in each prescription group. The number was not published, so we estimated the number of patients readmitted 365 days after discharge using the number of readmissions in each prescription group multiplied by the readmission proportion. In addition, we assessed the statistical significance of differences between the typical LAI group and the atypical LAI group. The χ^2^ test was performed with one degree of freedom, an upper limit of statistical significance of 5%, and a critical value of 3.84 for the readmission proportions of the typical LAI alone and atypical LAI alone groups. The policy research group used SPSS modeler 18.1, Microsoft Excel 2016, and Python3 in PyCharm for data analysis. We used the CHISQ.DIST.RT function in Microsoft Excel 2016 to calculate *P*‐values.

## Results

The data selection flow diagrams for Analysis 1 and Analysis 2 are shown in Figure 2a,b, respectively. The data included aggregated age and sex information. A total of 1 641 590 patients (718 010 men and 923 580 women) met all inclusion criteria for Analysis 1: 103 265 were aged <20 years, 463 048 were aged 20–39 years, 663 050 were aged 40–64 years, 181 284 were aged 65–74 years, and 230 943 were aged ≥75 years. Of these patients, 57 210 (3.5%) had received an LAI prescription: the first prescribed LAI was a typical LAI in 27 090 patients (47.4%) and an atypical LAI in 30 120 patients (52.6%). The LAI prescription proportion for each prefecture ranged from 2.0% to 6.8%; that is, there was a more than threefold variance among prefectures (Fig. 3).

**Figure 2:** Data selection flow diagrams. (a) Analysis 1. (b) Analysis 2. LAI, long‐acting antipsychotics injection; NDB, National Database of Health Insurance Claims and Specific Health Checkups of Japan.

RETRACTED

**Figure 3:** Long‐acting antipsychotic injection prescription proportions in Japan, by prefecture. Dark green: Top 10 prefectures. Light green: Medium‐ranked prefectures. White: Lowest 10 prefectures.

A total of 7907 patients (3975 men and 3932 women) met all criteria for Analysis 2: 71 were aged <20 years; 2456 were aged 20–39 years; 4505 were aged 40–64 years; 741 were aged 65–74 years; and 134 were aged ≥75 years. Among those who received an LAI prescription after discharge from a psychiatric facility, the readmission proportion within 365 days after discharge was as follows: 41.0% among all patients prescribed an LAI after discharge (*n* = 7907), 36.2% among patients prescribed only typical LAI (*n* = 210), 23.5% among patients prescribed only atypical LAI (*n* = 947), 43.9% among patients prescribed typical LAI and non‐LAI (*n* = 2496), 42.1% among patients prescribed atypical LAI and non‐LAI (*n* = 3946), and 59.6% among patients prescribed typical LAI, atypical LAI, and non‐LAI (*n* = 287) (Fig. 4). There were 21 patients who were prescribed typical LAI and atypical LAI in our dataset, but the readmission proportion could not be determined because NDB publication rules do not allow disclosure of data for any analysis when *n* < 10; thus, we concluded there were fewer than 10 patients in this group who were readmitted. The χ^2^ test revealed a significant difference between the group prescribed only atypical LAI and the group prescribed only typical LAI (χ^2^ = 14.48, *P* < 0.05, *P* = 0.00014).

**Figure 4:** Readmission proportions of outpatients with schizophrenia by LAI prescription classification. Yellow: prescribed LAI after discharge (*n* = 7907). Orange: prescribed only typical LAI (*n* = 210). Red: prescribed only atypical LAI (*n* = 947). Gray: prescribed typical and atypical LAI (*n* = 21) (unpublished percentage^1^). Light Blue: prescribed typical LAI and non‐LAI (*n* = 2496). Light Green: prescribed atypical LAI and non‐LAI (*n* = 3946). Navy: prescribed typical LAIs, atypical LAI, and non‐LAI (*n* = 287). Data for <10 patients is excluded from publication in accordance with NDB rules. ^1^The primary aim of this study was to describe the current status of LAI prescriptions in Japan, so we did not use a new‐user design or adjust for regional variations.

## Discussion

We analyzed the NDB data of patients with schizophrenia in Japan to investigate the LAI prescription proportion and the types of LAIs used among outpatients, as well as patient readmission proportions by type of LAI prescribed after discharge from a hospital.

RETRACTED

In previous large‐scale patient surveys conducted in other countries, LAI prescription proportions for patients with psychiatric disorders such as schizophrenia were approximately 21%–37%.^16^, ^17^, ^25^, ^26^ In the present study, LAIs were prescribed for only 3.5% of outpatients with schizophrenia receiving antipsychotics in Japan. This percentage is far lower than that in other countries, even when considering differences in study methodology for determining these proportions. Our results suggest that LAIs are prescribed less widely in Japan than in other countries. Fujii and Takahashi examined the reasons for avoiding atypical LAIs and compared their results with those of a similar study in Germany.^27^ They conducted a questionnaire survey of psychiatrists who had >3 years of experience and found that, compared with German psychiatrist, Japanese psychiatrists were more reluctant to prescribe LAIs. The greatest difference between Japanese and German psychiatrists was found in those with ‘little experience’ prescribing LAIs. Based on these results, Japanese psychiatrists may be caught in a vicious cycle where their limited experience prescribing LAIs leads to a negative attitude toward LAIs, which further restricts their experience with prescribing LAIs.

The LAI prescription proportion differed markedly (by more than threefold) among prefectures, ranging from 2.0% to 6.8%. This difference may have been due to (i) the prescribing trends of physicians in certain hospitals, which affects the region's prescribing trends and (ii) socioeconomic regional characteristics. LAIs are more likely to be prescribed in areas with poor access to health care than in those with good access to health care.

Few studies have compared prescription proportions between first‐generation (typical) LAIs and second‐generation (atypical) LAIs. In this study, the difference in LAI prescription proportions was small between conventional typical LAIs and the newer atypical LAIs, suggesting that in the short period since their introduction to Japan, atypical LAIs have been readily adopted in the Japanese clinical setting by physicians who already have experience with LAIs.

Analysis 2 determined the readmission proportions of patients with schizophrenia receiving LAIs after discharge from psychiatric facilities. The readmission proportion increased over time, reaching 41% at 365 days after discharge (Fig. 4). A previous study conducted in Japan estimated that the readmission proportion of patients with schizophrenia within 6 months after discharge was 30%.^28^, ^29^ In the present study, the readmission proportion at 6 months was approximately 27%, which is similar to or possibly lower than that in the previous report. However, it is difficult to compare these results because we did not analyze overall readmission proportions in this study. Kishimoto and colleagues reported in their 2013 meta‐analysis of randomized control trials that there was no significant difference in efficacy between LAIs and OAPs.^12^ More recently, they performed a meta‐analysis of cohort studies and demonstrated that LAIs decreased hospitalization rates significantly more than orally administered drugs.^13^ Although there are inconsistencies among previous meta‐analyses, we assume that our study's readmission proportions are closely aligned with those of this latter meta‐analysis because both used real‐world clinical data.

RETRACTED

We compared different types of LAIs and found that the readmission proportion (23.5%) was lower in patients prescribed atypical LAI alone than that in those prescribed typical LAI alone. This difference was significant and may reflect physicians' drug selection behaviors being influenced by the following factors: (i) atypical LAIs were introduced later than typical LAIs, so more physicians are likely to administer them in patients with a relatively short history of schizophrenia, (ii) atypical LAIs cause fewer side effects such as malaise than typical LAIs, leading to the higher continuation rate of atypical LAIs. We also found that the readmission proportion was the highest in patients who had been prescribed all three types of treatment (typical LAI, atypical LAI, and non‐LAI). This suggests that the physicians had been struggling to determine the best treatment for the patient and that atypical LAIs did not seem to be effective. Kishimoto and colleagues showed in their recent meta‐analysis of cohort studies that illness severity and/or chronicity was significantly greater in patients prescribed LAIs than in those prescribed OAPs.^13^ Another meta‐analysis of randomized controlled trials showed that the rate of treatment discontinuation and outcomes such as relapse and relapse‐related withdrawal were not significantly different between patients prescribed LAIs and those prescribed OAPs.^30^ These results may be due to patient selection bias. Further research is needed to understand the underlying factors, such as disease severity, contributing to the difference in readmission proportions between atypical and typical LAIs.

Of the patients who received LAIs within 90 days after discharge, 85.6% (*n* = 6750) received antipsychotics from multiple categories. This may be related to Japan's polypharmacy problem. For example, a 2016 REAP (Research on Asian Prescription Pattern) study examined the use of antipsychotics in patients with schizophrenia in Asian countries and found that the proportion of patients on a combination of two or more antipsychotics in Japan was 55.0%, higher than the proportions in other countries.^31^ However, the REAP study involved a limited number of facilities in specific areas of Japan. It is therefore difficult to compare the results of the REAP study with ours because of that study's limited generalizability and the presence of both inpatients and outpatients.

RETRACTED

A survey conducted by Okumura and colleagues investigated the administration of antipsychotic drugs to schizophrenic patients in Japan and used methods similar to those in the present study. They used data extracted from the NDB. After accounting for the number of generic names of antipsychotics prescribed in one month, more than 50.2% of all the outpatients with schizophrenia were prescribed more than one type of antipsychotic; however, the random sample was small.^32^ Previous extraction studies have shown that many outpatients with schizophrenia receive combination antipsychotic therapy, and the results of the present study show that this is also true for those using LAIs. Many studies have reported that antipsychotic polypharmacy is associated with increased risk of death.^33^, ^34^ Additionally, guidelines recommend avoiding polypharmacy with LAIs.^35^ As mentioned earlier, Japanese psychiatrists are known to be averse to prescribing LAIs because of their limited experience with LAIs. However, physicians should be encouraged to appropriately prescribe LAIs, for which monotherapy is recommended. This may contribute to decreasing the number of combinations of antipsychotics used by patients with schizophrenia.

To date, no published study has investigated the prescription proportion of each type of LAI nationwide in Japan using a large‐scale database such as the NDB. We believe that this study is of high clinical significance, particularly because the readmission proportion after discharge was analyzed over time. For policy making and future research, it is crucial to elucidate the current situation of healthcare in Japan from a clinical perspective.

This study has some limitations. First, the diagnosis records in the NDB are not definitive because this database is based on claims data. However, the likelihood of patients without schizophrenia receiving an LAI prescription is very low, so we assume the patients receiving LAI prescriptions were very likely patients with schizophrenia. On the other hand, inaccurate diagnosis may lead to overestimation of patients with schizophrenia prescribed OAPs. It is important to increase the diagnostic accuracy by adding parameters related to disease specificity in the future. Second, there is inherent selection bias because the current NDB is not representative of the data on patients not covered by this database (i.e. patients for whom all medical expenses were paid out of public funds other than health insurance), though a large majority of patients receive clinical care under the health insurance system. Third, the primary aim of this study was to investigate the current status of LAI prescriptions, so we did not adopt a new‐user design or adjust for regional variations. Finally, the dataset we used from the policy research group was limited to the period between 1 February 2015 and 31 March 2017. There may be selection bias and prevalent user bias, but our discussion was based on the notion that these biases did not critically influence our investigation of the current status of LAI prescriptions, which was the aim of this study.

RETRACTED

In Japan, where most of the population is covered by universal health insurance, we used NDB data to conduct this comprehensive study on the current status of LAI prescriptions and the outcomes of patients with LAI prescriptions. The study revealed that LAIs have not been widely adopted in Japan compared with other countries. The readmission proportion to psychiatric facilities was lower for patients with an atypical LAI prescription than with a typical LAI prescription.

## Disclosure statement

This study was a collaboration between the National Institute of Mental Health, National Center of Neurology and Psychiatry, and Otsuka Pharmaceutical Co., Ltd. We thank Otsuka Pharmaceutical Co., Ltd. for their generous financial support. MU, RO, and YY have no conflicts of interests to report. YK is a full‐time employee of Otsuka Pharmaceutical Co., Ltd.

## Author contributions

All authors conceived and designed the study. M.U. and Y.Y. analyzed the data. M.U. and R.O. drafted the article and wrote the manuscript. All authors critically reviewed the manuscript and approved the final version of this manuscript.

## Supporting information


**Table S1.** Supplementary table prepared in compliance with the International Society for Pharmaceutical Engineering guidelines.

**Table S2.** List of 29 antipsychotic drugs.
